The article "Personal Information Security Environment Monitoring and Law Protection Using Big Data Analysis" was retracted in 2023. Reasons: signs of a paper mill; suspected computer-generated content; unreliable results or conclusions; concerns about the data.

# Personal Information Security Environment Monitoring and Law Protection Using Big Data Analysis

**DOI:** 10.1155/2022/1558161

**Published:** 2022-10-07

**Authors:** Wei Zhu

**Affiliations:** Department of Law, East China Normal University, Shanghai 200241, China

## Abstract

This article explores the causes of the issues with personal data privacy and outlines the limitations of China's current legal framework. This article makes the argument that, in the information age, self-discipline and legal protection should be combined in order to safeguard personal information safety. It also makes specific recommendations for strengthening legal protection. This research also develops a data processing platform for data safety and privacy protection while studying the technology of data safety environment monitoring and privacy protection. This work develops optimization methodologies, such as dynamic privacy budget allocation, to increase the model's speed of convergence and the calibre of the generated data. It adjusts to various privacy and timeliness needs under the assumption that the objective of selective matching of private safety will be satisfied. According to the experimental findings, this algorithm's accuracy can reach 96.27%. This method enhances the model's speed of convergence and the calibre of the data created, and it addresses the flaw that the present data fusion publishing procedure cannot withstand the attack of background information. The study's findings can serve as a starting point for future work on data security and the protection of personal information.

## 1. Introduction

Big data is a significant symbol and resource in the contemporary environment of cross-integration and shared development of science and technology and industrial technology, and a great number of information databases are communicating with one another all over the world at an unprecedented scale and speed. The amount of data has increased as a result of the adoption and popularisation of cutting-edge technologies like cloud computing and IoT, ushering in the information era [1]. Due to the continuous progress of IT (Information Technology) [2, 3] and continuous use of data, data as an important strategic resource, implies great value. Enterprises, scientific and technological circles, and government departments began to effectively mine and use data in order to promote economic development and social progress. Data circulation is having a great impact on the world economy, politics, culture, society, military affairs, diplomacy, etc. With the introduction of IT, lifestyles have grown easier and more effective, and overall quality of life has increased dramatically. In order to respond to the establishment of new national strategic objectives and to promote innovation and business model reform with rapid social development and long-term economic growth, it is effective to combine data and personal information. Personal information is a crucial decision-making tool in the information society, and its importance to social progress cannot be overstated. The production and use of personal information has been facilitated by technological advancement, making the processing of personal information more convenient [4]. The development of big data technologies may lead to the creation of new privacy for information that was not previously thought to be private. The practise of gathering personal data is widespread, and the meaning attached to it is expanding. Additionally, it is simpler to obtain personal data. The importance of personal information has grown in this environment, making it necessary to find a solution to the paradox between protecting personal information and making use of it.

Under the operation of data technology, the ability of information collection and utilization has made a qualitative breakthrough, and our personal information is in danger of being illegally collected, used, and leaked in the special network environment. The phenomenon that personal information is infringed is more and more common. In the continuous processing and utilization of information, the subject of information is constantly infringed, and the personal privacy protection safety becomes increasingly serious. Common behaviors against personal information safety mainly include disclosure, illegal handling, and illegal use. In view of the increasingly serious problem of personal information leakage and abuse, most countries have promulgated and implemented personal data protection laws to provide law protection for personal information safety [5]. Most national and international legislations delimit the scope of personal data protection by identifiability and establish the right of personal information. In recent years, China has also accelerated the legislative progress of personal data protection and achieved remarkable results. However, in the new data age, the original protection and management methods are still facing great challenges [6]. Although the state pays more and more attention to the law personal privacy protection, the law personal privacy protection still lacks basic legal support, and the definition of personal information is not very clear and the concept is vague. The lack of relevant legislation leads to inadequate implementation of various measures and policies, which make the law protection of citizens' personal information, face great risks. In today's era, we must face up to the potential value of personal information, not abandon the collection and utilization of information in the name of protecting personal information, and constantly improve the personal privacy protection. Therefore, this paper discusses the law protection of personal details safety based on big data analysis.

Individual information safety requires personal information to be kept confidential, complete, and controllable without internal and external risks. The internal risk that threatens personal information safety mainly refers to the defects of IT itself, while the external risk mainly lies in people's illegal behavior. In the information age, various business models and social services driven by data have brought great convenience to people's daily life, but there are hidden dangers of personal privacy. This is mainly because the collected data more or less carry personal privacy data, but in the process of data collection, processing, and publishing, these privacy data have not been effectively protected [7]. Data typically includes a lot of very sensitive personal information about the user, including identity details, home address, medical information, salary information, travel itinerary details, and consumption logs. Without sufficient security measures, data release or use will result in major privacy disclosure, placing users' personal and property safety in grave danger. This study examines the primary privacy protection methods in order to address the issue of personal privacy data leaking. This study separates data safety into four categories based on the big data life cycle model: data storage safety, data access control, antibig data analysis and mining, and data publication privacy protection. It also examines and explores the safety technologies used at various phases. On the basis of this, a data processing platform for the protection of personal information is built. The following are the innovations of this paper:

1. This study conducts scientific and workable research to examine practical ways to enhance the law's protection of personal privacy and safety in China's information age based on the country's current legal framework. It also makes some recommendations for the development of China's personal data protection system. This essay outlines the fundamental legal safeguards for individual privacy in the information age. In a practical sense, this article offers personal information protection, which is helpful for fostering the growth of the data sector
2. This research suggests a hierarchical data fusion publishing method based on differential privacy protection in the personalised privacy protection data-publishing environment to address the issue of data privacy disclosure during the data fusion publishing process. This work designs three optimization strategies—dynamic privacy budget allocation, adaptive cropping threshold selection, and weight parameter clustering—to enhance the model's speed of convergence and the calibre of the data provided. It adjusts to various privacy and timeliness needs under the assumption that the objective of selective matching of private safety will be satisfied. This approach accelerates model convergence while resolving the issue that the current data fusion publishing mechanism cannot withstand the attack of background knowledge

## 2. Related Work

Individual information has the technical background of the Internet and the characteristics of personal privacy, so many studies also call it network privacy. Privacy protection technology, as one of the hottest directions in the field of information safety, provides technical guarantee for the privacy of data. At present, many scholars have studied the related content.

Gao believes that before collecting personal information legally, we should protect the safety of personal information, and personal information can either be immediately identified or all information identified as a specific individual will be delayed [8]. Yang and Qiao proposed that the role of industry self-discipline in the operation of big data should be developed, the role of endogenous regulation in self-discipline protection should be brought into play, and attention should be paid to the details of the combination of self-discipline protection and law, to increase its executive power and implementation [9]. Lei et al. pointed out that in the information age, due to the development of IT, personal information, in addition to personal data in the traditional sense, should also include the corresponding online personal information generated by its activities on the Internet, and the personal privacy protection constitutes law protection, the key to online privacy [10]. Zhang et al. discussed how to learn from the experience of foreign countries in dealing with personal data protection issues in legislation and specific systems under the interests of personal data protection and utilization, and how to build a personal data protection system in the network age challenge to respond [11]. Schadt explained the challenges and violations of citizens' personal data protection in the information society [12]. Chen pointed out that there are still major deficiencies in the current law personal privacy protection safety: lack of special legislation, and unclear legal provisions; multiple law enforcement, lax supervision; single legal remedy channels, high cost; information subjects and information managers' lack of personal legal awareness of information safety [13]. Liang and Xue pointed out that the promotion effect of unified legislation on personal data protection can be expected, so it is necessary to formulate a special personal data protection law to clarify the basic issues in the protection and utilization of personal information [14]. Kirkham et al. pointed out that data strengthens the association between personal details and personal privacy, and further distinguishes the difference between the two [15]. At the same time, the virtuality of data also affects the law personal privacy protection. Izanlou et al. conducted in-depth research on how to strengthen the personal privacy protection safety in the network age from the perspective of law, especially from the fields of legislative advice, law enforcement supervision, and judicial protection [16]. According to the type of data usage, Zhang et al. introduced three aspects: privacy protection research in static data release, privacy protection research in real-time data release, and privacy protection research in distributed learning [17]. Hwang et al. integrated the privacy protection mechanism with MapReduce distributed computing under the Hadoop platform, and proposed a distributed privacy protection algorithm for massive data [18]. Dong and Pi proposed a weight-attenuated streaming data publishing method by exploiting the data correlation in the data stream to reduce the consumption of the privacy budget [19]. Ambrosin et al. distorted the sensitive attributes in the original data by adding noise, while using the privacy budget to keep the data usable [20].

While traditional cryptography can theoretically ensure the security of data transport and storage, it restricts the sharing and deep mining of this data to some extent. Traditional privacy data publication approaches typically require the development of unique rules for each data set to deal with privacy aspects or to deal with high-dimensional data, which significantly reduces the usefulness of the data. As a result, this research suggests a GAN-based strategy for releasing differential privacy data (Generative Advanced Networks). A hierarchical data fusion publishing technique based on differential privacy protection is also proposed in this research for the personalised privacy-protected data publication environment. With this approach, the current data fusion publishing mechanism's weakness of being unable to fend off the attack of background knowledge is fixed, and the model's convergence speed and the calibre of the data it generates are both enhanced.

## 3. Methodology

### 3.1. Overview of Law Personal Privacy Protection Safety

Here are the following kinds of common personal information in society: (1) Identity personal information, (2) individual information of social relations, (3) individual information about behavior habits, and (4) Individual information of subjective tendency. In the data age, due to the continuous progress of IT, the commercial value of personal information is constantly improving, and personal information has become a kind of “commodity” [21]. However, its material value is also realized through the information subject, and the material benefits mainly come from the specific object pointed by the spiritual world, that is, the information subject, and the materialization form that respects and safeguards the basic spiritual interests of human beings. The internal meaning and external definition of personal information determine the scope of powers and responsibilities that should be protected when the personal data protection law is enacted [22]. However, there are laws and administrative rules in related fields, as well as the pertinent provisions of the Tort Liability Law, Criminal Law, and other departmental laws to ensure the safety of personal information. At the moment, China has not promulgated any special laws to regulate the collection, analysis, and use of personal information. The study of personal information security in this work is based on a limited definition of information security that emphasises the privacy of individual data. In order to determine which personal information needs to be protected and which behaviors violate the rights and interests, it is necessary to understand the basic content, legal meaning, and legal attributes of personal information, as well as to define it reasonably in terms of its actual scope [23]. The use of IT broadens the concept of conventional personal information, and the line separating personal data protection rapidly blurs. This not only causes the right to safeguard personal information to become less clear, but also makes it more difficult to share and use personal information. If we do not move quickly to preserve personal information and if we cannot tightly control and deal with the illegal acts that breach citizens' privacy, then not only will the information collector's privacy be invaded but also his personal property will sustain significant financial losses. Although China's Internet industry self-discipline is still in the early stages of development, there is still a sizable gap in how it addresses the protection of individual privacy in the digital age.

### 3.2. Law Protection Measures of Personal Information

Personal information security issues are getting more and more complex under the current IT landscape. This paper proposes various countermeasures to enhance law personal privacy protection in the information age based on an in-depth examination of the subject. They are as follows:

1. *Define the basic legal category of personal information protection law*. The definition of the scope of personal information should be based on a set of judgment rules instead of a simple judgment standard. It has certain advantages to divide “personally identifiable information” into identified information and identifiable information. These two kinds of information can be reasonably protected, and various risk factors can be organically integrated to clearly divide their risk levels. Sensitive information should be protected and general information should be used reasonably. At the same time, set the time limit for the storage of personal information. Under reasonable circumstances, the information must be deleted when the storage time reaches the prescribed time limit, and the data controller must delete the personal information when the relevant personal information is used and kept by others without reasonable reasons. To clarify the rights and obligations between the information subject and the user, the data manager should use personal information in a legal way, follow its basic principles and requirements, and actively fulfill the obligation to protect personal information safety. On the legislative level, it puts forward clear and strict requirements for private enterprises to ensure the safety of personal information. That is, all social organizations that join the industry self-discipline must use, collect, and process personal information in strict accordance with industry rules and legislative principles. If you violate the above rules, you will not only be punished by the industry rules but also be punished by law
2. *Clarify the rights and obligations of information managers*. Authorize the Ministry of Legislation and Industry to manage self-regulatory organizations and norms, endow them with corresponding law enforcement powers, and formulate clear terms of reference and law enforcement procedures. When members of self-regulatory organizations violate the rules of self-regulation, the supervisory organization has the right to impose corresponding penalties on them. Due to the weak ability of social autonomy and the lack of self-discipline tradition and concept, the value of self-discipline in the industry will be lost if the state only supervises it. Therefore, it is necessary to set up a special industry supervision organization
3. *Clarify the basic concepts and principles of the personal data protection law*. We should determine the value concept of paying equal attention to personal information personality right and development and utilization right, and take this as the guiding ideology to design and formulate personal data protection rules. Self-discipline can only be regarded as complying with the legal provisions and the requirements of personal data protection through the approval of censors. Whether the censors can exercise their duties in an orderly manner is the key to whether the combination of legislative protection and self-discipline protection can play a great role, and it is also the important core of whether self-discipline norms can effectively protect personal information safety in the network age. At the same time, it is necessary to publicize the knowledge of network safety and enhance people's awareness of risk prevention. Starting with the people themselves, enhancing the right awareness of information subjects will protect personal information more effectively
4. *Create the safety net that will protect and allow you to use your personal information*. Establishing a safeguard mechanism for the use and protection of personal information is important to ensure the security of such data. Included are the mechanisms for personal data protection's implementation, alleviation, supervision, and self-discipline. To preserve the user's right to know about personal information, the information collector, for instance, should disclose the goal and purpose of the information up front and inform the recipient of the information. Likewise, information gatherers should consciously uphold their duty to disclose and take appropriate action when a user's personal information is violated, disclosed, or its intended use is altered while being processed. These mechanisms should be able to ensure that the relevant legal subjects of personal data protection can collect, use, and process personal information in strict accordance with the relevant laws. When the corresponding illegal infringement occurs, it can be found in time and dealt with according to law, so as to promote the full use of personal information and ensure the smooth realization of citizens' legitimate rights and interests of personal information. Through these mechanisms, the collection, utilization, and processing of personal information can be guaranteed legally and reasonably
5. *Combination of legislative protection and self-discipline protection*. The combination of legislative protection and self-discipline protection can make up for the lack of self-discipline in the industry to a certain extent, strengthen the enforcement of self-discipline norms, and appropriately increase the supervision of public power, which is more conducive to protecting the legitimate rights and interests of personal information subjects. Personal data protection is a very complicated problem in the information age. The combination of legislative protection and self-discipline protection can improve the stability and lag of the law, and give full play to the inherent regulatory advantages of self-discipline protection.

After a series of external safeguard measures, such as enacting laws, strengthening supervision, and improving relief mechanism, the government, industry organizations, and information collectors should also strengthen their awareness of personal information safety protection. Generally speaking, we should take the legislative value of the correct legal system of personal information as the guide and formulate specific norms, ensure that personal information is used more rationally on the basis of personal interests, and promote economic development and social progress.

### 3.3. Data Safety and Privacy Protection Data Processing Platform

Differential privacy protection model, with strict privacy definition and ability to fend against background knowledge intrusion by introducing noise to the alteration of the original data set or its statistical findings, it achieves the goal of privacy protection. This technique makes sure that altering a record in any data set will not have an impact on the query's output result. The standard differential privacy protection method is enhanced in this research, and a platform for data processing that protects privacy while storing data is created. This paper combines differential privacy and GAN to publish privacy data to ensure the confidentiality and availability of the five elements of information safety while also enabling the privacy protection data publishing method to be applied to more data sets and maintain high data availability with a small privacy budget. The data distributed storage system, data processing, authorization, and authentication make up the majority of the data safety storage and privacy protection data processing platform. The Hadoop and Spark distributed storage frameworks are used by the data storage system, and the distributed computing framework enables parallel processing and quick processing of large amounts of data. The user's access permissions are audited using the key management server, and different rights are granted based on the user's role. In this system, identity authentication and privacy protection distributed training make up the secure distributed training. In order to protect the privacy of the results, the noise generated by the differential privacy mechanism is added to the total results in the stage of publishing the private results. In addition, this paper fuzzifies the tuples in the candidate list to eliminate the delay of data release, that is, to ensure that all tuples can be released in time. At the same time, fuzzy processing can solve the balance between data utility and privacy protection, and improve the practicality and privacy safety of published data.  Figure 1 shows the architecture diagram of data processing platform.

CDP (Centralized Differential Privacy) gives two data sets *D* and *D*′, which are identical or at most different by one record. Given the random algorithm *A*, Ran(*A*) represents the range of *A*, and *S* is a subset of Ran(*A*). If *A* satisfies Formula (1), then algorithm *A* satisfies *ε* − CDP.

(1) $$\begin{array}{c} \text{Pr}\left[A\left(D\right)\in S\right]\leq e^{\varepsilon }\times \text{Pr}\left[A\left(D^{\prime }\right)\in S\right], \end{array}$$

where the probability Pr[·] represents the probability of the algorithm, which is determined by the algorithm *A*; *ε* is the privacy budget, which indicates the privacy protection degree of algorithm *A*, and usually takes the values of 0.01, 0.1, or 1, etc. The smaller the value of *ε*, the higher the privacy protection degree of *A*, and the worse the practicality of data.

For any function *f* : *D*⟶*R*^*d*^, if the algorithm *Y* satisfies the Formula (2), it is said that *Y* satisfies *ε*− differential privacy.

(2) $$\begin{array}{c} Y\left(D\right)=f\left(D\right)+\langle {\text{Lap}}_{1}\left(\Delta f/\varepsilon \right),\cdots ,{\text{Lap}}_{d}\left(\Delta f/\varepsilon \right)\rangle , \end{array}$$

where the function Lap_1_(Δ*f*/*ε*)(1 ≤ *i* ≤ *d*) represents the Laplace density function; Δ*f* = max_*D*_1_,*D*_1__|*f*(*D*_1_) − *f*(*D*_2_)| is the query sensitivity of the function *f*(*D*). *D*_1_ and *D*_2_ are sibling data sets; *d* is the query dimension. For any function *f* : *D*⟶*R*^*d*^, the global sensitivity of function *f* is

(3) $$\begin{array}{c} \Delta f=\max{\left\|f\left(D_{1}\right)-f\left(D_{2}\right)\right\|}_{p}. \end{array}$$

Among them, *D*_1_ and *D*_2_ differ by at most one record; *R* represents the mapped real number space; *d* represents the query dimension of the function; *p* indicates the *L*_*p*_ distance used to measure Δ*f*, which is usually measured by *L*_1_.

Similar groups are fused and averaged in the data statistical publication process, and the average of fused groups is used to replace the original statistical findings of groups in order to address the issue of outliers in the data publishing process, which increases the danger of privacy disclosure. Namely:

(4) $$\begin{array}{c} C_{\text{gd}}^{\prime }=\frac{C_{i}+C_{i+1}}{2}. \end{array}$$

Among them, the judgment of outliers is

(5) $$\begin{array}{c} S_{i-1}<<S_{i}\&\&S_{i+1}<<S_{i}. \end{array}$$

Then add noise interference on the basis of average.

The generating network does not need to explicitly establish the concept density function, that is, it learns the complex features in high-dimensional data and can output the synthetic data, which is very close to the original data. GAN is mainly inspired by binary zero-sum game and consists of a pair of opposing models. The generator *G* and the discriminator D. The following minimax game issue can be used to define the objective function of GAN:

(6) $$\begin{array}{c} \underset{G}{\min}\underset{D}{\min}V\left(D,G\right)=E_{x-\text{Pdate}}\left[\log D_{w}\left(x\right)\right]+E_{z-p_{z}\left(z\right)}\left[\log\left(1-D_{w}\left(G_{\theta }\left(z\right)\right)\right)\right], \end{array}$$

where *G* is the generator; *D* is a discriminator; *E* is asking for expectations; *x* is a real data sample; *z* is a noise sample; *G*(*z*) is the data generated by the generator. The loss functions of generator and discriminator are as follows:

(7) $$\begin{array}{c} \arg\min-D_{w}\left(G_{\theta }\left(z\right)\right),\\ \arg\min D_{w}\left(G_{\theta }\left(z\right)\right)-D_{w}\left(z\right)+\lambda {\left({\left\|\nabla_{\overset{⌢}{x}}D_{w}\left(\overset{⌢}{x}\right)\right\|}_{2}-1\right)}^{2}. \end{array}$$

Among them:

(8) $$\begin{array}{c} \overset{⌢}{x}=\varepsilon x+\left(1-\varepsilon \right)G_{\theta }\left(z\right), \end{array}$$

where *ε* is a random number that obeys [0, 1] uniform distribution. The gradient penalty might hasten the algorithm's convergence by acting as the function's regularisation term.

The algorithm's objective is to introduce noise through “target disturbance” into the polynomial coefficients of the model's objective function. The optimization process can offer privacy constraints, enabling differential privacy protection for the data set's components. Let the database *D* in regression analysis contain *nd* + 1 dimensional tuples

(9) $$\begin{array}{c} \left\{t_{i}\left|i=1,\cdots ,n\right.\right\}. \end{array}$$

Among them:

(10) $$\begin{array}{c} t_{i}=\left(x_{i},y_{j}\right)=\left(x_{i1},x_{i2},\cdots ,x_{\text{id}},y_{i}\right),\\ \sqrt{\overset{d}{\underset{i=1}{\sum }}x_{\text{id}}^{2}}\leq 1. \end{array}$$

The regression model function *f* takes *x*_*i*_(*i* = 1, ⋯, *n*) and the parameter vector *w* as input, and outputs the predicted value *y*_*i*_^∗^(*i* = 1, ⋯, *n*) of *y*_*i*_(*i* = 1, ⋯, *n*). Let the polynomial of ***£*** be expressed as:

(11) $$\begin{array}{c} £\left(f,D\right)=\overset{J}{\underset{j=0}{\sum }}\underset{\varphi \in \Phi_{j}}{\sum }\overset{n}{\underset{i=1}{\sum }}\lambda_{\varphi_{i}}\varphi \left(w\right). \end{array}$$

The solution to the problem is the parameter *w* that minimizes ***£***. The function mechanism takes *D*, *f*, and ***£*** as inputs, and then adds Laplace noise to the coefficient *λ*_*φ*_*i*__ of ***£*** to obtain the noised objective function **£**^∗^. Finally, solve the parameter vector *w*^∗^ that makes **£**^∗^ reach the minimum value, which is the return value of the algorithm. Using *w*^∗^ as the input to *f* for prediction will not reveal the information of {*t*_*i*_|*i* = 1, ⋯, *n*} in the database *D*.

In order not to cause additional privacy loss, this method designs three optional noise attenuation functions without touching the original privacy data, so that the noise scale *σ* is periodically updated in units of training rounds. Exponential Noise Attenuation:

(12) $$\begin{array}{c} \sigma_{t}=\sigma_{0}e^{-\text{kt}}. \end{array}$$

Among them, *σ*_0_ is the initial noise size; *t* is the current number of training rounds; *k*(*k* > 0) is the decay rate. Periodic Noise Attenuation:

(13) $$\begin{array}{c} \sigma_{t}=\sigma_{0}*k^{\left[t/\text{period}\right]}, \end{array}$$

where the parameter period is the update period of the noise. Polynomial Noise Attenuation:

(14) $$\begin{array}{c} \sigma_{t}=\left(\sigma_{0}-\sigma_{\text{end}}\right)*{\left(1-t/\text{period}\right)}^{k}+\sigma_{\text{end}}, \end{array}$$

where *σ*_end_(*σ*_end_ < *σ*_0_) is the final size of the noise. When the number of training rounds is t < period, the noise is continuously reduced to *σ*_end_; when it is t > period, the noise remains unchanged at *σ*_end_.

In this study, the data processing platform is used to build a noninteractive differential privacy protection data processing module. This module uses Spark to safeguard the privacy of the data and primarily gathers and saves the original data. In order to prevent hostile participants from destroying the noise scale, the merging function converts the original ciphertext calculation function and average noise adding function into a cloud function. Along with improving safety, the merge function also improves model framework structure, decreases participant workload, and accomplishes a better integration of various technologies. In order to calculate the global weight parameters, the server first decrypts the gradient aggregation value using the secret share that the user has uploaded. The server is in charge of securely aggregating gradient ciphertext. The cloud server is also in charge of examining each user's gradient ciphertext signature in order to confirm the veracity of their identity. The gradients of most bias parameters in the GAN model are close to 0, however the gradients of weight parameters are significantly bigger than 0 and very dissimilar from one another. In light of this, this research proposes the clustering of weight parameters 2. The weight parameters are classified into various classes using the density-clustering algorithm, and the classification gradient cutting is performed for each class of parameters 1. All bias parameters are still uniformly cut by gradient. The data is stored using a distributed data storage system, and the data analysts read the data from the cluster, process it with the aid of the platform, and report back to the data analysts the findings of their processing. The data processing platform's deployment diagram is shown in Figure 2.

Hierarchical data fusion publishing is mainly composed of multiple data sources, trusted agents, and query users. (1) Multiple data source owners fuse their own data through classification fusion algorithm. (2) Carry out personalised differential privacy protection on the fused data, and set reasonable different privacy budget parameters. (3) When the user inquires, the pseudonym mechanism is used to protect the privacy of the user.

## 4. Result Analysis and Discussion

To assess the effectiveness of the suggested method for data publishing, experimental simulations are carried out in this section on the privacy processing effectiveness and information loss of published data. Protection of privacy and data security A cluster of six machines running Windows and equipped with 32G of memory makes up the data processing platform. The other hosts are slave compute nodes, with one host acting as the master node. Built atop the Hadoop foundation is the Spark platform. All of the experimental algorithms were developed in MATLAB. The inaccuracy rate of released data can be used to gauge the classification standard of user level. The privacy budget parameter is set to 0.1 if the data user anticipates receiving data with a query result error rate of less than 1%; it is set to 0.005 if they anticipate receiving data with an error rate of between 10% and 20%. As a result, in this experiment, the privacy budget parameters (0.001,0.1) are chosen, and users are rated based on their values. Prior to doing the experiments on MNIST, Poker Hands, and Transactions, the discriminator and generator are developed. The generator's noise dimension is 100, with each dimension having a maximum value of [-1,1]. The inception scores for real data and artificial data are displayed in Table 1.

Comparing different methods, it can be seen that the optimization strategy in this paper improves the quality of generated data, and at the same time, it can better balance the quality and privacy of generated data.

Streaming data is divided using the sliding window module. The data in the window is continuously updated when new data is entered, and the window advances when the amount of data reaches the window size. Statistics are performed in accordance with categories and data clustering analysis is performed using the fractal clustering module. In reality, privacy concerns are frequently complex, and the goal of privacy protection cannot be fulfilled by a single differential privacy protection paradigm. Multiple differential privacy protection models might be required in this situation to safeguard the output results' confidentiality. Serial combinability and parallel combinability, two significant combinatorial properties of differential privacy, can guarantee that the combined models of several differential privacy models still satisfy differential privacy. Calculating the privacy loss is the key to understanding the differential privacy data publishing algorithm's safety. To make sure that the data produced by the generator satisfies the requirements for differential privacy, the differential privacy protection is applied to the discriminator in this study. However, the loss of privacy is unrelated to the volume of synthesised data because GAN can continue to do so indefinitely. The insertion, deletion, and change of data can all be handled effectively using this procedure. Additionally, since no phoney tuples or sounds are produced and all the data may be broadcast in real time, the published data's veracity is guaranteed.  Figure 3 displays the algorithm's training loss.

This paper verifies and analyzes the relationship between privacy disclosure risk and published data dimension. Among them, privacy disclosure risk method is used to measure the risk of privacy disclosure.  Figure 4 shows the impact of increasing data dimensions on privacy risk.

In the execution of differential privacy, function sensitivity is a crucial factor. However, the sensitivity would be considerably impacted by the calculation that was outsourced to the cloud server and the aggregation method employed. As a result, while applying functions, care should be taken to consider their sensitivity. The approximate ideal clipping threshold for each parameter in each training cycle is first calculated using its gradient, and the parameters with comparable thresholds are then pooled into a sort of postclipping gradient, to which noise is added. By using this method of classification and clipping, it is possible to avoid overnoising some parameters and slowing the model's convergence rate. The quality of the obtained data is improved in the latter training phase as a result of the noise scale dynamically decreasing during the training process. On the MNIST data set, Figure 5 compares the runtime efficiencies of several algorithms.  Figure 6 compares the running effectiveness of various algorithms on the CelebA dataset.

In constraint spectrum clustering, the constraint information displayed by labels can greatly improve the clustering accuracy. To ensure fairness, all constraint spectrum clusters adopt consistent constraint information matrix and consistent landmark points. After clustering, the original large data set has been divided into different small data sets. Then, the clustered small datasets are sorted, difference sets, and grouped. The categorization accuracy of data produced using various techniques on standard data sets are displayed in Table 2.  Table 3 displays the data clustering accuracy for data produced using various techniques on benchmark data sets.

The analysis shows that this method can balance the usability and privacy of the generated data.

Data safety and privacy protection, the data processing platform realizes privacy protection of sensitive data by intervening Laplacian noise with different values. This algorithm is based on the set user levels and privacy budgets corresponding to user levels. Generally speaking, higher privacy budget value means lower noise level and lower privacy protection level, that is, better retention of mining function. The trusted agent stores the user level to the query server. According to the query level of platform users, different privacy budgets are set, and data sets with corresponding privacy protection degree are published. The accuracy test results of the algorithm are shown in Figure 7.

According to the experimental findings, this algorithm's accuracy can reach 96.27%. This approach can successfully satisfy the privacy publishing requirements of dynamic data while also guaranteeing the accessibility of published data. The extensive analysis of the algorithm on data sets demonstrates that it can produce high-quality data with no loss of privacy, making it suitable for a range of data research activities.

## 5. Conclusion

Under the current background, personal information implies great economic value. To tap its value, the development and utilization of personal information has become a fact and a trend. Nowadays, with the data mining and utilization, the contradiction between personal details safety and information freedom has become increasingly prominent. How to balance the relationship between the two has become an unavoidable problem in legislation and concrete system construction. In the era of commercialization of personal information, law protection should play a guiding and stimulating role in addition to the mandatory and prohibitive provisions, so that information controllers can take the initiative to protect personal information safety, thus achieving the purpose of better protecting personal information from the source. Based on this, this paper puts forward that to protect personal information safety in the information age; we should choose the combination of self-discipline protection and law protection, and puts forward specific suggestions to improve law protection.

The main technologies for data security and privacy protection are thoroughly examined in this study, and a data processing platform for these purposes is built. This research suggests a hierarchical data fusion publishing technique based on differential privacy preservation in the personalised privacy-preserving data publication environment. The present data fusion publishing process cannot withstand the background knowledge assault; however, our method fixes that issue. In addition, this study offers optimization strategies including dynamic privacy budget allocation to enhance the model's speed of convergence and the calibre of the generated data. It adjusts to various privacy and timeliness needs under the assumption that the objective of selective matching of private safety will be satisfied. According to the experimental findings, this algorithm's accuracy can reach 96.27%. This approach can successfully satisfy the privacy publishing requirements of dynamic data while also guaranteeing the accessibility of published data. With this approach, both the model's convergence rate and the calibre of the generated data are improved. However, this paper's consideration of personal data protection is still in its early stages. More and more in-depth research is required in order to strengthen the personal data protection system overall in the modern day.

## Figures and Tables

**Figure 1:** Architecture diagram of data processing platform.

**Figure 2:** Deployment diagram of data processing platform.

**Figure 3:** Loss of algorithm training.

**Figure 4:** Impact of increasing data dimension on privacy risk.

**Figure 5:** Comparison of running efficiency of different algorithms on MNIST dataset.

**Figure 6:** Comparison of running efficiency of different algorithms on transactions dataset.

**Figure 7:** Accuracy test results of the algorithm.

**Table 1:** Inception scores of real data and synthetic data.

Data set	Algorithm	*n*(×10^4^)	(*ε*, *δ*)	Scores
MNIST	Real data	6	—	9.95 ± 0.02
	Methods of this paper	6	—	9.53 ± 0.02
	DPGAN	6	(4, 10^−5^)	9.12 ± 0.02
	WGAN-GP	6	—	8.51 ± 0.03

Poker hand	Real data	3	—	4.89 ± 0.01
	Methods of this paper	3	—	4.34 ± 0.01
	DPGAN	3	(15, 10^−5^)	3.15 ± 0.01
	WGAN-GP	3	—	2.86 ± 0.01

**Table 2:** Classification accuracy of data generated by different methods on standard datasets.

Data set	Real data	Paper method	DPGAN	WGAN-GP
MNIST	99.81%	97.48%	84.05%	84.37%
Transactions	95.72%	92.36%	87.46%	80.49%
Poker hand	89.46%	88.51%	71.14%	81.71%

**Table 3:** Clustering accuracy of data generated by different methods on standard datasets.

Data set	Real data	Paper method	DPGAN	WGAN-GP
MNIST	99.4%	97.87%	88.51%	81.29%
Transactions	93.2%	90.68%	84.65%	82.47%
Poker hand	88.5%	86.91%	85.32%	80.64%

## Data Availability

The data used to support the findings of this study are available from the corresponding author upon request.
